# Study on the Mechanism of Action of Paclitaxel-Loaded Polylactic-co-glycolic Acid Nanoparticles in Non-Small-Cell Lung Carcinoma Cells

**DOI:** 10.1155/2022/8524951

**Published:** 2022-04-06

**Authors:** Yangsong Zuo, Wenyi Shen, Lili Wang, Chengshi Wang, Juan Pu

**Affiliations:** ^1^Department of Aspiration Medicine, Lianshui County People's Hospital, Lianshui, Huaian 223400, Jiangsu, China; ^2^Department of Radiotherapy, Lianshui County People's Hospital, Lianshui, Huaian 223400, Jiangsu, China

## Abstract

**Objective:**

To study effective carriers that can enhance the antitumor effect of paclitaxel (PTX).

**Methods:**

PTX-loaded polylactic-co-glycolic acid (PLGA) nanoparticles (NPs) (PTX-PLGA NPs), constructed using the emulsification solvent evaporation method, were characterized by scanning electron microscopy and dynamic light scattering. Non-small-cell lung carcinoma (NSCLC) cells were divided into the dimethyl sulfoxide (DMSO) group, PLGA NPs group, PTX group, and PTX-PLGA NPs group. Cell viability was detected by 3-(4,5-dimethylthiazol-2-yl)-2,5-diphenyltetrazolium bromide (MTT), cell apoptosis was determined by flow cytometry, and cell migration and invasion were assessed using Transwell assay.

**Results:**

PTX-PLGA NPs were smooth in the surface and spherical in shape, with a particle size of 268 ± 1.3 nm. Both PTX and PTX-PLGA NPs could effectively inhibit the activity of A549 and H1650 cells. At 12 and 24 h, PTX-PLGA NPs presented weaker inhibition on the activity of NSCLC cells than PTX, but at 48 and 72 h, PTX-PLGA NPs presented stronger inhibition. Compared with PTX, PTX-PLGA NPs were more effective in enhancing apoptosis and inhibiting migration and invasion of NSCLC cells.

**Conclusion:**

With good sustained release and the ability to promote cellular uptake, PTX-PLGA NPs can strongly inhibit the malignant activities of NSCLC cells, which can be used as a promising drug carrier.

## 1. Introduction

Non-small-cell lung carcinoma (NSCLC) is the primary subtype of lung cancer, the most common cause of death [1]. NSCLC can be classified as either adenocarcinoma, squamous cell carcinoma, or large cell carcinoma. Adenocarcinoma usually originates from alveolar cells located in the small airway epithelium, while squamous cell carcinoma arises from the cells of the airway epithelium, and large cell carcinoma is composed of large cells with rich cytoplasm and large nucleoli [2]. Currently, chemotherapy, including paclitaxel (PTX), is the mainstay of treatment for NSCLC [3]. Exploring novel and effective PTX-based strategies for NSCLC is important for the treatment of patients with NSCLC.

PTX, extracted from Taxus brevifolia (Pacific yew), is a tricyclic diterpene [4]. Its antitumor ability is based on its promotion of tubulin assembly and inhibition of tubulin depolymerization [5]. Currently, solvents such as ethanol and polyoxyethylene castor oil are frequently used with PTX to overcome the water solubility of PTX [6]. As an effective treatment, solvent-bound PTX has been widely used in the treatment of NSCLC [7]. However, this therapy still has the disadvantages of potential toxicity and hypersensitivity [8].

The use of liposomes or polymers can improve the efficiency of drug delivery and the efficacy of therapy [9]. For example, Yu et al. [10] applied maytansine-loaded zein nanoparticles (NPs) to the treatment of NSCLC and found that the NPs could greatly enhance the maytansine uptake in NSCLC cells, thus directly enhancing the antitumor effect of maytansine in NSCLC. Lee et al. [11] found that NPs controlled the release of Adriamycin and celecoxib in acidic tumor microenvironments and enhanced the inhibitory effect of CD44 on the malignant phenotype of NSCLC. Additionally, Elbatanony et al. [12] demonstrated that polylactic-co-glycolic acid- (PLAG-) loaded afatinib was beneficial to enhance the efficacy of afatinib in NSCLC cells in vitro. Binding PTX to NPs can facilitate drug penetration into tumor microenvironments, thus increasing the binding affinity of drugs to cancer cells [13]. PLGA NPs are increasingly used in anticancer therapy and early diagnosis of cancer [14]. Mittal et al. [15] reported that PTX-loaded PLGA NPs (PTX-PLGA NPs) could overcome the limitations of current solvents. Moreover, Luiz et al. [16] revealed that folic acid-modified PLGA NPs loaded with PTX could significantly enhance the uptake of PTX by ovarian cancer cells and strengthen the antitumor effect of PTX.

At present, there are few studies on the treatment of NSCLC with PTX-PLGA nanoparticles. Therefore, PTX-PLGA NPs were prepared in this study to investigate the in vitro therapeutic effect of the composite particles in NSCLC, exploring their potential for the treatment of this disease.

## 2. Materials and Methods

### 2.1. Preparation and Characterization of PTX-PLGA NPs

PTX and PLGA were dissolved in dichloromethane (DCM) solution and gradually added to 1% polyethylene (PE) aqueous solution after full dissolution. The solution was placed in ice for ultrasonic oscillation for 5 min, followed by 4 h of stirring at normal pressure and 30 min of centrifugation at 2.3 × 10^4^ r/min for precipitate collection. The precipitate was then cleaned, frozen, and dried to obtain the PTX-PLGA NPs. Finally, the morphology of PTX-PLGA NPs was observed by scanning electron microscopy (SEM; Geneline Bioscience, Beijing, China), and the potential and particle size were detected by dynamic light scattering (DLS).

### 2.2. In Vitro Release Kinetics

Phosphate-buffered saline (PBS; Shanghai Aladdin Biochemical Technology Co., Ltd., Shanghai, China, P196987-500 mL) solution containing PTX-PLGA NPs were oscillated in a constant temperature shaker at 37°Cin the dark. On days 1–24, the solution was centrifuged at 17,000xg at 4°C for 15 min to collect the supernatant. Finally, the concentration of PTX in the supernatant was determined using an ultraviolet (UV) spectrophotometer (Shanghai Aiyan Biotechnology Co., Ltd., Shanghai, China, A30221), and the in vitro release profile was drawn.

### 2.3. Cell Viability

Eight wells were selected from each of the three 12-well plates to inoculate A549/H1650 cell lines (ATCC, USA). Each cell line was seeded into four wells of the plate and named as the dimethyl sulfoxide (DMSO) group, PLGA NPs group, PTX group, and PTX-PLGA NPs group, respectively. At 24, 48, and 72 h, a 3-(4,5-dimethylthiazol-2-yl)-2,5-diphenyltetrazolium bromide (MTT) reagent was added to one plate, following the instructions provided with the kit (Solarbio, China). The optical density of each sample at 570 nm was then measured by spectrophotometry, and the cell viability was assessed.

### 2.4. Apoptosis

The cells were prepared as suspensions and treated with ethanol (volume fraction: 70%) at 0°Cfor 24 h. Apoptosis was determined using a corresponding fluorescein isothiocyanate (FITC)/Annexin V kit (BD Biosciences, USA), and cell apoptosis rate was analyzed using CellQuest acquisition software (BD Biosciences, USA).

### 2.5. Cell Migration and Invasion

A Transwell chamber (upper compartment planted with cells) was subjected to 24 h incubation (37°C, 5% CO_2_), followed by removal of the fluid in the upper compartment and removal of the cells on the microporous membrane. Cells on the other side of the membrane were treated with 4% paraformaldehyde (PFA) for 15−20 min, followed by 15−20 min of staining with crystal violet (Beijing Solarbio Science & Technology Co., Ltd., Beijing, China, G1061-500) and cleaning of the chamber. Finally, images of the cell migration were collected under an optical microscope and the number of cells was counted. The experiment was repeated three times. Cell invasion was detected in the same manner as above after laying an 8% matrix gel (Shanghai Yanhui Biotechnology Co., Ltd., Shanghai, China, 354234) on the plate, and the number of cells per well was changed to 5 × 10^4^.

### 2.6. Statistical Analysis

GraphPad Prism 6 (GraphPad Software, San Diego, USA) was used for statistical analysis and image rendering. The experimental results of the two cell lines were expressed as the mean ± SD; one-way analysis of variance (ANOVA) was used for comparison of experimental results among multiple groups, and Dunnett's *t*-test was used for post hoc pairwise comparison. P values less than 0.05 were considered to indicate statistical significance within the 95% confidence interval.

## 3. Results and Discussion

### 3.1. Characterization of PTX-PLGA NPs

In this study, PTX-PLGA NPs were constructed by the emulsification solvent evaporation method (ESEM), and the NPs were characterized by using SEM and DLS (Figure 1). PTX-PLGA NPs were spherical, with a smooth surface, uniform particle size (268 ± 1.3 nm), good sphericity, and Zeta potential of −13.1 ± 0.3 mv.

### 3.2. In Vitro Release Kinetics of PTX-PLGA NPs

The drug loading and entrapment efficiency of PTX-PLGA NPs were 9.39% and 82.52%, respectively. As shown in Figure 2, the cumulative release rate of PTX-PLGA NPs reached approximately 50% in the first 10 days and then gradually slowed down, reaching 66.11 ± 1.39% after 3 weeks. Therefore, PTX-PLGA NPs show favorable sustained release.

### 3.3. Effect of PTX-PLGA NPs on Viability of NSCLC Cells

NSCLC cells were divided into the DMSO group, PLGA-NPs group, PTX group, and PTX-PLGA NPs group, and the cell viability of each group was detected. As shown in Figure 3, PTX and PTX-PLGA NPs could effectively inhibit the activity of A549 and H1650 cells, and the inhibitory effect of PTX-PLGA NPs on NSCLC cells at 24 h was lower than that of PTX at 24 h and stronger than that of PTX at 48 h and 72 h.

### 3.4. Effect of PTX-PLGA NPs on Apoptosis of NSCLC Cells

The apoptosis process of cancer cells was significantly inhibited during their life cycle. In this study, it was found that both PTX and PTX-PLGA NPs can induce apoptosis of NSCLC cells, and PTX-PLGA NPs can induce apoptosis of NSCLC cells more effectively than PTX (Figures 4 and 5).

### 3.5. Effect of PTX-PLGA NPs on Metastasis of NSCLC Cells

In this paper, Transwell assay was used to detect the migration and invasion ability of NSCLC cell lines A549 and H1650. As shown in Figure 6, both PTX and PTX-PLGA NPs could inhibit the migration and invasion of NSCLC cells, and PTX-PLGA NPs had a stronger inhibitory effect.

The above results suggest that PTX-PLGA NPs can more effectively inhibit the viability, migration, and invasion of NSCLC cells and promoted apoptosis compared with the solvent-based PTX.

### 3.6. Discussion

Drug delivery to tumor cells requires both the stability of the drug in the blood circulation and its sufficient accumulation in the tumor. In addition, in order to maximize the effect of drug therapy, drug permeability, affinity with tumor cells, and release kinetics should be in an ideal state [17]. A growing number of studies have shown that NPs are beneficial to drug delivery and biocompatibility of drugs, which can improve the drug effect [18–24]. PLGA, which is copolymerized from lactic acid monomers and glycolic acid monomers, has favorable biocompatibility and degradability, so it is extensively applied in drug delivery systems [25]. Increasing evidence suggests that PLGA NPs are reliable drug carriers in drug delivery. Nigam et al. [26] demonstrated that lamotrigine-loaded PLGA NPs could greatly alleviate neuropathic pain and improve the efficiency of intranasal administration of lamotrigine. Esfandyari-Manesh et al. [27] showed that PEG-modified PLGA NPs could load imatinib effectively and that the composite particles could effectively target atherosclerosis. Moreover, PLGA NPs functionalized with PEG and maleimide can also be used as mucoadhesive carriers for intravesicaldrug delivery [28].

We used the ESEM to construct PTX-PLGA NPs and found via SEM and DLS that their potential and particle size were −13.1 ± 0.3 mv and 268 ± 1.3 nm, respectively. The results of in vitro release kinetics curves showed that the combination of PTX and PLGA NPs can significantly enhance the release kinetics of PTX. According to the cytotoxicity test, PTX significantly inhibited the growth of NSCLC cells at 24 h, but at 48 and 72 h, the growth activity recovered and PTX did not exert further inhibition; however, PTX-PLGA NPs exerted consistent inhibition on cell growth and activity during the abovementioned time period. The results indicate that PTX-PLGA NPs exhibited an obvious sustained-release effect during drug delivery, providing a stable guarantee for the antitumor effect of PTX. Jiménez-López et al. [29] revealed that the application of PTX-loaded PLGA NPs to immunocompetent mice could significantly suppress the tumor volume, showing a certain therapeutic effect in vivo.

Inactive apoptosis of cancer cells results in low mortality of malignant cells [30]. Many previous studies [31–34] have shown that PTX can induce apoptosis of cancer cells to a certain extent. Yuan et al. [35] also reported that the PTX delivery system based on PLGA-Tween 80 copolymer can significantly induce apoptosis of A549 cells and thus play a therapeutic role in vitro, which is similar to our research results. The results of this study demonstrated that PTX-PLGA NPs had a stronger induction effect on cell apoptosis than PTX. In addition to inactive apoptosis, both migration and invasion are typical malignant activities of cancer cells. In this study, PTX could inhibit the malignant migration and invasion of NSCLC cells, but its inhibitory effect was weaker than that of PTX-PLGA NPs. Therefore, PTX-PLGA NPs are superior to PTX in inhibiting the malignant activities of NSCLC cells. This study also has certain novelty. First, we analyzed the characterization of PTX-PLGA NPs by SEM and DLS and confirmed their good drug-loading properties by in vitro release kinetic curves. Second, the therapeutic mechanism of PTX-PLGA NPs in NSCLC cells was analyzed from the dimensions of cell viability, apoptosis, migration, and invasion.

## 4. Conclusion

In conclusion, given the effective inhibitory effect of PTX-PLGA NPs on the malignant behavior of NSCLC cells, as well as a good sustained release effect and a high promotion of cellular uptake, PTX-PLGA NPs can be used as a promising drug carrier that is worthy of promotion and application in the research and treatment of NSCLC.

## Figures and Tables

**Figure 1:** Characteristics of PTX-PLGA NPs. (a, b) Potential and particle size of PTX-PLGA NPs (−13.1 ± 0.3 mv and 268 ± 1.3 nm, respectively). (c) Morphology of PTX-PLGA NPs. PTX-PLGA NPs: paclitaxel-loaded polylactic-co-glycolic acid nanoparticles.

**Figure 2:** In vitro release kinetics of PTX-PLGA NPs. The cumulative release rate of PTX-PLGA NPs reached approximately 50% in the first 10 days and then gradually slowed down, reaching 66.11 ± 1.39% after 3 weeks. PTX-PLGA NPs: paclitaxel-loaded polylactic-co-glycolic acid nanoparticles.

**Figure 3:** Effect of PTX-PLGA NPs on cell viability. (a) At 24 h, PTX-PLGA NPs presented weaker inhibition on the viability of A549 cells compared to PTX, but at 48 and 72 h, PTX-PLGA NPs presented stronger inhibition than PTX. (b) At 24 h, PTX-PLGA NPs presented weaker inhibition on the viability of H1650 cells than PTX, but at 48 and 72 h, PTX-PLGA NPs presented stronger inhibition than PTX. ^∗^*P* < 0.05, ^∗∗^*P* < 0.01, and ^∗∗∗^*P* < 0.001. PTX: paclitaxel; PLGA-NPs: polylactic-co-glycolic acid nanoparticles; PTX-PLGA-NPs: paclitaxel-loaded polylactic-co-glycolic acid nanoparticles.

**Figure 4:** Apoptosis assay (scatter diagram) measured by flow cytometry.

**Figure 5:** Effect of PTX-PLGA NPs on cell apoptosis. (a) PTX-PLGA NPs can more significantly promote the apoptosis of A549 cells than PTX. (b) PTX-PLGA NPs can more significantly promote the apoptosis of H1650 cells than PTX. ^∗^*P* < 0.05, ^∗∗^*P* < 0.01. PTX: paclitaxel; PLGA-NPs: polylactic-co-glycolic acid nanoparticles; PTX-PLGA-NPs: paclitaxel-loaded polylactic-co-glycolic acid nanoparticles.

**Figure 6:** Effect of PTX-PLGA NPs on cell migration and invasion. (a) PTX-PLGA NPs can more significantly promote the migration and invasion of A549 cells than PTX. (b) PTX-PLGA NPs can more significantly promote the migration and invasion of H1650 cells than PTX. ^∗^*P* < 0.05. PTX: paclitaxel; PLGA-NPs: polylactic-co-glycolic acid nanoparticles; PTX-PLGA-NPs: paclitaxel-loaded polylactic-co-glycolic acid nanoparticles.

## Data Availability

The labeled datasets used to support the findings of this study are available from the corresponding author upon request.
